# TRIM11 overexpression promotes proliferation, migration and invasion of lung cancer cells

This article has been retracted.

**DOI:** 10.1186/s13046-016-0379-y

**Published:** 2016-06-21

**Authors:** Xiaolin Wang, Weiping Shi, Hongcan Shi, Shichun Lu, Kang Wang, Chao Sun, Jiansheng He, Weiguo Jin, Xiaoxia Lv, Hui Zou, Yusheng Shu

**Affiliations:** Department of Thoracic Surgery, Northern Jiangsu People’s Hospital and Clinical Medical College of Yangzhou University Yangzhou, No. 98 Nantong West Road, Yangzhou, 225001 People’s Republic of China

**Keywords:** TRIM11, Lung cancer, PI3K/AKT, Migration, Invasion

## Abstract

**Background:**

Tripartite Motif Containing 11 (TRIM11), a member of TRIM proteins, is overexpressed in high-grade gliomas and plays an oncogenic function in glioma biology. However, little is known about the role of TRIM11 in lung cancer.

**Methods:**

We analyzed TRIM11 mRNA expression in lung cancer tissues and adjacent non-neoplastic tissues by real-time PCR. We then explored the function of TRIM11 in lung cancer cells by small interfering RNA-mediated downregulation of this protein followed by analyses of cell proliferation, migration and invasion.

**Results:**

TRIM11 was highly expressed in lung cancer tissues and lung cancer cell lines. The higher expression of TRIM11 was correlated with the poorer prognosis of patients. Suppressing of TRIM11 expression in lung cancer cells with higher expression of TRIM11 (A549 and NCI-H446 cells) significantly reduced cell growth, motility and invasiveness. We further demonstrated that knockdown of TRIM11 affected the expression of cell proliferation-related proteins (Cyclin D1 and PCNA), and epithelial-mesenchymal transformation-related proteins (VEGF, MMP-2, MMP-9, Twist1, Snail and E-cadherin). The activity of ERK and PI3K/AKT was also suppressed in TRIM11 knocked down cells. Further experiments in lung cells with lower expression of TRIM11 (NCI-H460 and NCI-H1975 cells) with AKT inhibitor suggested that TRIM11 may promote cell motility and invasiveness through AKT pathway.

**Conclusions:**

Our results indicate that TRIM11 acts as an oncogene in lung cancer through promoting cell growth, migration and invasion. Our findings may have important implication for the detection and treatment of lung cancer.

**Electronic supplementary material:**

The online version of this article (doi:10.1186/s13046-016-0379-y) contains supplementary material, which is available to authorized users.

## Background

Lung cancer is the most frequently diagnosed malignancy. It is the leading cause of cancer death with over 1 million death annually in the world [1]. Non-small cell lung carcinoma (NSCLC) is the most frequently occurring of lung cancer and accounts for approximately 85 % of lung cancer [1]. NSCLC includes adenocarcinoma (ADC), squamous cell carcinoma (SCC), large cell carcinoma (LCC) and others [2]. Despite recent advances in diagnosis and treatment, the prognosis of lung cancer is still poor [3]. Therefore, a better understanding of which pathways or proteins are active in lung tumor progression will contribute to the development of early detection and targeted therapy for lung cancer [4–6].

Tripartite Motif Containing (TRIM) proteins are characterized by the presence of tripartite motif, which is composed of a RING domain, 1 or 2 B-box motifs and a coiled-coil region (RBCC) [7]. Most members of TRIM proteins, including TRIM11 could be defined as E3 ubiquitin ligases. Besides RBCC domain, TRIM11 contains a PRY domain and a SPRY domain. TRIM11 is thought to destabilize Humanin (24-amino-acid neuroprotective peptide) [8], activator-recruited cofactor 105-kDa component (ARC105) [9], PAX6 (a member of the paired-box family of transcription factors) [10] and PHOX2B (a paired box homeodomain transcription factor) [11]. Earlier studies on TRIM11 have revealed its roles in nervous system function and development [8, 10, 11]. Recently, TRIM11 expression was found elevated in high-grade gliomas and it may exert an oncogenic function in glioma biology [12]. Other members of TRIM proteins, such as TRIM25 [13] and TRIM59 [14], have been reported to be upregulated in lung cancer, while TRIM16 [15] and TRIM31 [16] were found decreased in NSCLC. However, few investigation has been performed to test the expression and functions of TRIM11 in lung cancer.

In this study, TRIM11 expression was frequently higher in lung cancer tissues than corresponding adjacent non-neoplastic tissues. We investigated whether TRIM11 regulated cell proliferation and metastasis of lung cancer. Our study showed that TRIM11 promoted cell migration and invasion by activating the PI3K/AKT signal pathway. Our findings suggest that TRIM11 is a new potential target in lung cancer.

## Methods

### Samples

120 patients with lung cancer undergoing surgical resection at Department of Thoracic Surgery, Northern Jiangsu People’s Hospital (Yangzhou, China) were enrolled in this study. The age of enrolled patients was between 34 and 72 (median 56) years. 63 participants (52.5 %) were male and 57 (47.5 %) were female. Primary lung cancer tissues were collected from all enrolled patients, while adjacent non-cancerous tissues were obtained from 35 patients of the enrolled patients. The follow-up lasted 5 years. The study was reviewed and approved by Research Ethic Committee in Northern Jiangsu People’s Hospital (Yangzhou, China). Written informed consent was obtained from all patients.

### RNA isolation and real-time PCR

Total RNA from tissues and cells was extracted using Trizol (Invitrogen, Carlsbad, CA, USA) according to the manufacturer’s protocol. The residual DNA was removed by treating with DNase I (Roche, Indianapolis, IN, USA). Real-time PCR was used to evaluate TRIM11 mRNA levels. Total RNA (2 μg) was reverse-transcribed to cDNA with M-MLV Reverse Transcriptase Kit (Thermo Fisher, Rockford, IL, USA). The resulted cDNA was used for real-time PCR with SYBR Green qPCR Master Mix (Thermo Fisher) on ABI 7300 system (Applied Biosystem, Foster City, CA, USA) following manufacturer’s instruction. The relative TRIM11 mRNA levels were calculated by normalization to GAPDH mRNA levels. The PCR primers were as follows: TRIM11 forward, 5’- CACCTAAGCTGCACAGTTCC-3’; TRIM11 reverse, 5’- GGCTGCCTCCTAATTCTTCC -3’; GAPDH forward, 5’-CACCCACTCCTCCACCTTTG-3’; GAPDH reverse, 5’- CCACCACCCTGTTGCTGTAG -3’.

### Western blotting

Frozen tissue sample (about 0.1 g) was ground into powder using liquid nitrogen. Protein was extracted from frozen tissue powder and cultured cells by using RIPA lysis buffer (JRDUN Biotech., Shanghai, China) with fresh-added proteinase inhibitor cocktail (Sigma, St. Louis, MO, USA) on ice for 15 min and centrifuged at 12,000 rpm for 20 min. Protein concentrations were determined using a bicinchoninic acid kit (Thermo Fisher). For Western blotting analysis, lysates (30 μg/well) were subjected to SDS-PAGE and transferred onto nitrocellulose filter membranes. After blocking in 5 % skim milk at room temperature for 30 min, the membranes were incubated with primary antibodies overnight at 4 °C. Horseradish peroxidase conjugated secondary antibodies were subsequently used. Signals were detected using chemiluminescenct substrate (ECL; Bio-Rad, Richmond, CA, USA) and exposed to X-ray film. The results were scanned and analyzed using Image J software (http://rsb.info.nih.gov/ij/, Bethesda, MD, USA). Antibodies against anti-TRIM11, proliferating cell nuclear antigen (PCNA), vascular endothelial growth factor (VEGF), matrix metalloproteinase (MMP)-2, MMP-9, Twist1, PI3K and p-PI3K were from Abcam (Cambridge, MA, USA). Antibodies against CyclinD1, Snail, E-cadherin (CDH1), AKT, p-AKT, ERK, p-ERK and GAPDH Cell Signaling Technology (Danvers, MA, USA).

### Cell culture

Human lung adenocarcinoma cell lines A549, NCI-H1975 and PC-9, human large cell lung carcinoma cell lines NCI-H460, small cell lung cancer cell line NCI-H446 and human embryo lung fibroblasts MRC-5 were obtained from cell bank of Shanghai Biology Institute, Chinese Academy of Science (Shanghai, China). The lung cancer cell lines were cultured in RPMI 1640 medium (Invitrogen; Carlsbad, CA, USA). MRC-5 cells were maintained in Eagle’s Minimum Essential Medium (EMEM). Both medium were supplemented with 10 % fetal bovine serum (FBS; Gibco, Los Angeles, CA, USA), 1 % penicillin/streptomycin and 2 mM L-glutamine. All cell lines were cultured in at 37 °C, 5 % CO_2_.

### Knockdown of TRIM11 expression by small interference RNA (siRNA) transfection

Three siRNA targeting human TRIM11 mRNA (siRNA1, 5’- CAGAAGUUGUGCCUAUGGA -3’; siRNA2, 5’- GCUAUUACAAUUCCUCGGA -3’; and siRNA3, 5’- CUAUUCAUCUUUCCCGAGA -3’) and a non-specific control siRNA sequence (NC) were synthesized by Genepharma (Shanghai, China) and transfected into A549 and NCI-H446 cells with Lipofectamine 2000 (Invitrogen, Carlsbad, CA, USA) per the manufacture’s instruction. Real-time PCR and Western blot analysis were performed at 48 h after transfection to assess knockdown efficiency.

### Construction of TRIM11 lentivirus

Full-length human TRIM11 was cloned into the pLVX-AcGFP1-C1 (Clontech, Palo Alto, CA, USA). Lentiviral constructs of pLVX-AcGFP1-C1 empty vector or pLVX-AcGFP1-C1-TRIM11 were cotransfected with viral packaging plasmids (psPAX2 and pMD2.G) into 293 T cells with Lipofectamine 2000. At 48 h post transfection, viral supernatant was collected to infected NCI-H460 and NCI-1975 cells.

### Cell proliferation assay

A proliferation assay was carried out using Cell Counting Kit-8 (CCK-8, Dojindo Laboratories, Japan) according to the manufacturer’s protocol [17]. Briefly, 2000 cells/well were seeded into 96-well plates and transfected with indicated siRNA. The cells were cultured for 0, 24, 48 and 72 h, then 10 μL CCK-8 reagent was added to each well and the cells were incubated at 37 °C for 1 h. The absorbance was recorded at 450 nm with a microplate reader (Bio-Rad).

### Transwell migration and invasion assays

Cell migration was assayed using Transwell with 8-μm-pore filters (Corning; New York, NY, USA) as previously described [5]. Cells were treated with the desired siRNA or expression virus. At 24 h after treatment, cells were trypsinized, resuspended in serum-free RPMI1640 medium and placed in the upper chamber (5 × 10^4^ cells/well) and treated with MK-2206 (Merck, Germany) or DMSO (Sigma). Then RPMI 1640 medium supplemented with 10 % FBS was added to the lower chamber. Non-migrating cells in the upper chamber were completely removed with a cotton swab 24 h later. Migrated cells were stained with 0.5 % crystal violet and counted in five random fields.

Cell invasion assays were also performed in the same condition expect that the upper chamber was pre-coated with Matrigel (BD Biosciences, Franklin Lakes, NJ, USA).

### Statistical analysis

All values are expressed as the mean ± SD. Statistical analysis was tested using Graphpad Prism (Graphpad Software, San Diego, CA, USA). For comparison between groups, statistical differences were tested with one-way analysis of variance (ANOVA), followed by a Sidak’s test for multiple comparisons. Fisher’s exact test was carried out to evaluate the relationship between TRIM11 mRNA expression and clinicopathological features. Kaplan-Meier survival curves were generated and compared by log-rank analysis. *P* < 0.05 was considered significantly different.

## Results

### TRIM11 was highly expressed in lung cancer tissue

We re-analyzed TRIM11 expression on lung cancer cohort from The Cancer Genome Atlas project (TCGA, https://tcga-data.nci.nih.gov/tcga/), including 58 normal tissue samples and 488 tumor tissue samples. The results showed that TRIM11 was highly expressed in tumor tissues compared with normal tissues (Fig. 1a, *P* < 0.0001).

**Fig. 1:** TRIM11 expression in lung cancer tissues **a** Analysis of TRIM11 expression in lung cancer tissues (*n* = 488) and normal tissues (*n* = 58) in TCGA dataset. **b** TRIM11 mRNA levels in lung cancer and normal tissues from patients admitted to Department of Thoracic Surgery, Northern Jiangsu People’s Hospital were determined by real-time PCR, with GAPDH as a control. **c** Kaplan-Meier survival analysis of 120 lung cancer patients revealed the correlation between TRIM11 expression and prognosis

We then detected TRIM11 mRNA levels in lung cancer (*n* = 120) and adjacent normal tissues (*n* = 35) by quantitative real-time PCR. As shown in Fig. 1b, TRIM11 expression was significantly higher in lung cancer tissues than that in normal tissues (*P* < 0.0001).

Then, according to the TRIM11 expression in tumor tissues, the 120 lung cancer patients were classified into two groups: TRIM11 higher group (*n* = 60) and lower group (*n* = 60). Then, the association between TRRM11 expression and patients’ features was analyzed by Fisher’s exact test. As shown in Table 1, TRIM11 expression was significantly correlated with tumor size, TNM stage and lymph node metastasis. While, no correlation was observed between TRIM11 expression level and age, gender or tumor type. Kaplan-Meier analysis showed that the overall survival time of patients with higher TRIM11 expression (median survival time: 27 months) was significantly shorter than those with lower TRIM11 expression (median survival time: 54 months, Fig. 1c, *P* < 0.01). Our data demonstrated that TRIM11 was overexpressed in lung cancer tissues and its expression was closely related with poor survival of patients with lung cancer.

**Table 1:** Correlation of TRIM11 expression with patients’ features

Variables	All cases	TRIM11	mRNA	
		Low (*n* = 60)	High (*n* = 60)	*P* value
Age at surgery				
< 55	48	25	23	0.8523
> =55	72	35	37	
Gender				
Male	63	31	32	1.0000
Female	57	29	28	
Tumor type				
SCC	52	31	21	0.1112
ADC	34	14	20	
LCC	13	8	5	
SCLC	21	7	14	
Tumor size				
< 5 cm	49	32	17	0.0090**
> =5 cm	71	28	43	
TNM stage				
I + II	55	36	19	0.0032**
III	65	24	41	
Lymphnode metastasis				
Absent	66	41	25	0.0057**
Present	54	19	35	

*Abbreviations*: *SCC* squamous cell carcinoma, *ADC* adenocarcinoma, *LCC* large cell carcinoma, *SCLC* small cell lung cancer

**P < 0.01

### TRIM11 mRNA expression was inhibited in cells transfected with the TRIM11 siRNAs

TRIM11 mRNA expression was determined in 5 lung cancer cell lines (A549, NCI-H446, NCI-H1975, NCI-H460 and PC-9) and 1 human embryo lung fibroblast cell line (MRC-5). As shown in Fig. 2a, TRIM11 mRNA level was higher in most lung cancer cell lines than in MRC-5 cells. We observed similar results in the protein levels of TRIM11 (Fig. 2b).

**Fig. 2:** TRIM11 was highly expressed in lung cancer cells and its expression was suppressed by TRIM11 siRNA transfection. **a** Real-time PCR analysis for the TRIM11 mRNA expression level in 5 lung cancer cell lines (A549, NCI-H446, NCI-H1975, NCI-H460 and PC-9) and 1 human embryo lung fibroblast cell line (MRC-5). **P < 0.01 and ***P < 0.001 versus MRC-5 cells. **b** TRIM11 protein expression was determined by Western blot. Quantification (*right panel*) based on at least 3 independent experiments was made by normalizing against GAPDH levels. **P < 0.01 and ***P < 0.001 versus MRC-5 cells. **c** Real-time PCR analysis showed the efficiency of TRIM11 knockdown in A549 and NCI-H446 cells. WT: wild-type cells. NC: control siRNA-transfected cells. siRNA1, 2 and 3: TRIM11 siRNA1, 2 or 3-transfected cells. ***P < 0.001 versus NC. **d** The protein levels of TRIM11 were determined by Western blot and GAPDH was used as an internal control. Quantification (*right panel*) was shown. ***P < 0.001 versus NC

In order to understand the functional relevance of TRIM11 expression in lung cancer progression, TRIM11 knock-down cell lines were generated by siRNA transfection. We selected two target cell lines, A549 and NCI-H446, which showed high levels of TRIM11 expression. As shown in Fig. 2c, control scrambled siRNA (NC) had no effects on TRIM11 mRNA expression compared with wild-type (WT) cells. TRIM11 siRNAs (siRNA1, siRNA2 and siRNA3) significantly inhibited TRIM11 mRNA expression compared to cells transfected with NC in both cell lines. siRNA3 had the best inhibition effect on TRIM11 mRNA expression. Western blot analysis was performed to confirm that TRIM11 protein expression was efficiently inhibited by siRNA3 transfection in both cell lines (Fig. 2d). Therefore, siRNA3 was used in all the subsequent experiments.

### Inhibition of TRIM11 expression decreased cell proliferation

CCK-8 assay was performed to determine whether TRIM11 plays a role in the growth of lung cancer cells. Cell growth of A549, NCI-H446 (Fig. 3a and b), NCI-H460 and NCI-H1975 (Additional file 1: Figure S1) cells was obviously repressed at 48 h and 72 h after TRIM11 expression was inhibited by siRNA3 transfection. On the contrary, cell growth of two lung cancer cell lines with low levels of TRIM11 expression (NCI-H460 and NCI-H1975 cells) was significantly increased by TRIM11 overexpression (Additional file 1: Figure S2).

**Fig. 3:** Knockdown of TRIM11 reduced the proliferation of lung cancer cells. **a**, **b** CCK-8 assay results of A549 and NCI- H446 cells at 0 h, 24 h, 48 h and 72 h after TRIM11 expression was inhibited by siRNA3 transfection. **c**, **d** Expression of PCNA and Cyclin D1 was evaluated by Western blot. Quantification (*bottom panel*) based on at least 3 independent experiments was shown. ***P < 0.001 versus NC

The protein levels of proliferation regulation proteins, PCNA and Cyclin D1, were evaluated by Western blot. The levels of PCNA and Cyclin D1 were reduced in TRIM11 knockdown cells (Fig. 3c and d). These results suggested that inhibition of TRIM11 expression inhibited cell proliferation in lung cancer cells.

### Suppressing of TRIM11 expression inhibited the motility and invasiveness of lung cancer cells

The ability of cancer cells to undergo migration and invasion allows them to spread with the tissues and metastasize to distant organs [18]. To investigate the function of TRIM11 in the metastasis, the effects of TRIM11 on the migrated and invasive ability of lung cancer cells were assessed by Transwell assay. As shown in Fig. 4a and b, silencing of TRIM11 in A549 and NCI-H446 cells caused a significant reduction in cell migration and cell invasion.

**Fig. 4:** Knockdown of TRIM11 inhibited the motility and invasiveness of lung cancer cells. **a** Migration assay was performed on wild-type (WT) cells, cells transfected with control siRNA (NC) and cells transfected with TRIM11 siRNA3 (siRNA3). Representative images (*left panel*) and quantitative results (*right panel*) were shown. **b** Invasion assay was carried out. **c**, **d** Expression of metastasis-related proteins was evaluated by Western blot. e *P < 0.05, **P < 0.01 and ***P < 0.001 versus NC

Moreover, epithelial-mesenchymal transformation (EMT) is critical for metastasis of cancer cells [19]. We then detected the protein levels of metastasis and EMT related proteins by Western blot (Fig 4c and d). The protein levels of VEGF, MMP-2, MMP-9, Snail and Twist1 were significantly down-regulated in A549 and NCI-H446 cells with TRIM11 knockdown, while the main factor of EMT, E-cadherin (CDH1) was significantly increased in TRIM11 knockdown cells. These data suggested an inhibitory role of TRIM11 on EMT and lung cancer metastasis.

### Silencing of TRIM11 repressed the activation of AKT pathway in lung cancer cells

Extracellular signal-regulated kinases (ERKs) [20] and PI3K/AKT [21] pathways, which are key signaling pathways involved in cell growth and migration, are frequently overactivated in tumor cells. Knockdown of TRIM11 in glioblastoma multiforme cells suppressed the activity of ERK pathway, while had no effects on PI3K/AKT activity [12]. To explore the effect of TRIM11 on PI3K/AKT and ERK pathways in lung cancer cells, phosphorylation of PI3K, AKT and ERK was determined by Western blot. As shown in Fig. 5, transfection of TRIM11 siRNA in lung cancer cells significantly reduced the phosphorylation of PI3K, AKT and ERK.

**Fig. 5:** Knockdown of TRIM11 inhibited the activation of PI3K/AKT and ERK pathways in lung cancer cells. Total protein and phosphorylation of PI3K, AKT and ERK was evaluated by western blot in A549 **a** and NCI-H446 cells **b**. **P < 0.01 and ***P < 0.001 versus NC

To further confirm the involvement of PI3K/AKT signaling, an AKT inhibitor (MK-2206) was used. NCI-H460 and NCI-H1975 cells, which showed low levels of TRIM11 expression, was overexpressed with TRIM11 and treated with MK-2206. Cell migration and invasion was then evaluated by Transwell assays (Fig. 6). Cell migration and invasion of lung cells was significantly enhanced by TRIM11 overexpression, but suppressed by MK-2206 treatment. More importantly, the promotion effects of TRIM11 overexpression on cell migration and invasion were weakened by MK-2206 exposure. These data indicated that TRIM11 may promote cell migration and invasion partially by activating PI3K/AKT pathway.

**Fig. 6:** Ectopic expression of TRIM11 impaired the effects of AKT inhibitor on the migration and invasion of lung cancer cells. **a**, **b** NCI-H460 and NCI-1975 cells were infected with control virus (Vector) or TRIM11 virus, and migration and invasion assay were performed in the present of either DMSO or AKT inhibitor (MK-2206, 2 μM). MK-2206 was dissolved in DMSO as a 10 mM stock solution. Thus, 0.02 % DMSO was used as negative control. ***P < 0.001 versus Vector + DMSO; ###*P* < 0.001 versus TRIM11 + DMSO; $$$*P* < 0.001 versus Vector + MK-2206

## Discussion

The altered expression of TRIM proteins has been reported in a variety of human cancers, including lung cancer [13–16]. Di, K. et al. demostrated diagnostic and prognostic value of TRIM11 in gliomas [12]. However, the expression and function of TRIM11 in lung cancer has been poorly characterized. Here, by analyzing online available dataset (Fig. 1a), we found that TRIM11 mRNA was elevated in lung cancer tissues, which was confirmed by real-time PCR analysis on 120 patients admitted at Department of Thoracic Surgery, Northern Jiangsu People’s Hospital (Fig. 1b). Fisher’s exact tests (Table 1) and Kaplan-Meier survival curves (Fig. 1c) demonstrated the strong association between TRIM11 expression and tumor size, TNM stage, lymph node metastasis, as well as overall survival of lung cancer patients. Thus, TRIM11 may serve as a useful diagnosis and prognosis marker for lung cancer although further in-depth clinical study is needed.

Then we investigated the functions of TRIM11 in lung cancer. The in vitro experiments demonstrated that inhibition of TRIM11 expression in lung cancer cells with higher expression of TRIM11 (A549 and NCI-H446 cells) suppressed cell growth (Fig. 3), migration (Fig. 4a) and invasion (Fig. 4b). On the contrary, ectopic expression of TRIM11 in in lung cells with lower expression of TRIM11 (NCI-H460 and NCI-H1975 cells) had inverse effects (Additional file 1: Figure S2 and Fig. 6). These data suggest that TRIM11 may play an oncogenic role by promoting the proliferation, migration and invasion of lung cancer cells. Our results of in vitro experiments were consistent to our clinical observation that high expression of TRIM11 associated with lymph node metastasis and tumor size. Furthermore, cancer cells gain migratory and invasive properties through the process of EMT [22]. Functional loss of E-cadherin has been considered as a key event during the process of EMT [23]. Twist1 and Snail can repress the expression of E-cadherin, and has been regarded as EMT-inducers [24]. VEGF [25] and MMP-2/9 [26] are well-known to play an important role in tumor metastasis. Here, knockdown of TRIM11 decreased the expression of metastasis (VEGF, MMP-2 and MMP-9) and EMT-related proteins (Twist1 and Snail), while increased the expression of E-cadherin. Our data suggested that TRIM11 siRNA may inhibit lung cell invasion via suppressing EMT.

Further, in addition to cellular phenotype, we tried to investigate the molecular mechanism through which TRIM11 works as an oncogene in lung cancer. ERK and PI3K/AKT pathways can promote cell growth and metastasis [27, 28]. Both ERK [20] and PI3K/AKT [21] pathways are frequently over-activated in various tumor types. Di, K. et al. found that knockdown of TRIM11 in glioblastoma multiforme cells had no effects on PI3K/AKT activity, but suppressed ERK activity [12]. In the current study, we found a notable decrease of ERK and PI3K/AKT activation (Fig. 5) in TRIM11 knocked down lung cancer cells. The discrepancy of data and the previous study [12] could be due to the different cell types used. Accumulating evidence points to the important role of cell motility and invasion in cancer progression and metastasis [29]. Phosphorylation levels of AKT was found to be associated with the invasion and metastasis of NSCLC [30]. In the present study, TRIM11 overexpression can promote the PI3K/AKT pathway (Additional file 1: Figure S2). The promotion effects of TRIM11 overexpression on cell migration and invasion were significantly weakened by the exposure of AKT inhibitor, MK-2206 (Fig. 6), which suggested that TRIM11 might promote cell migration and invasion partially by activating AKT pathway. Thus, we speculated that elevated TRIM11 will facilitate the development and invasive property of lung cancer through AKT pathways. However, the mechanisms are needed to be further elucidated in detail.

## Conclusions

In summary, increased expression of TRIM11 was noted in lung cancer tissues. TRIM11 functions as an oncogene in lung cancer through promoting cell proliferation, migration and invasion. Moreover, we demonstrated that TRIM11 may modulate PI3K/AKT pathway (Fig. 7). Considering that TRIM11 expression level was associated with patients’ overall survival, TRIM11 may be a new potential target in lung cancer treatment.

**Fig. 7:** Schematic representation of the biologic role of TRIM11 in lung cancer. TRIM11 may act as an oncogene lung cancer by promoting cell proliferation, migration and invasion. TRIM11 may modulate PI3K/AKT pathway

## Abbreviations

ARC105, activator-recruited cofactor 105-kDa component; CCK-8, Cell Counting Kit-8; EMEM, Eagle’s Minimum Essential Medium; EMT, epithelial-mesenchymal transformation; ERKs, extracellular signal-regulated kinases; FBS, fetal bovine serum; MMP, matrix metalloproteinase; NSCLC, non-small cell lung carcinoma; PCNA, proliferating cell nuclear antigen; TCGA, The Cancer Genome Atlas project; TIRM, Tripartite Motif Containing; VEGF, vascular endothelial growth factor.

## Additional file

Additional file 1: Figure S1. Knockdown of TRIM11 reduced the proliferation of NCI-H460 and NCI-H1975 cells. **Figure S2.** Effects of TRIM11 overexpression on cell proliferation. (DOCX 884 kb)

## References

[1] Torre LA, Bray F, Siegel RL, Ferlay J, Lortet-Tieulent J, Jemal A (2015). Global cancer statistics, 2012. CA Cancer J Clin.

[2] Koudelakova V, Kneblova M, Trojanec R, Drabek J, Hajduch M (2013). Non-small cell lung cancer--genetic predictors. Biomed Pap Med Fac Univ Palacky Olomouc Czech Repub.

[3] Longo-Sorbello GS, Chen B, Budak-Alpdogan T, Bertino JR (2007). Role of pemetrexed in non-small cell lung cancer. Cancer Invest.

[4] Zhou N, Wang H, Liu H, Xue H, Lin F, Meng X (2015). Mta1-upregulated epcam is associated with metastatic behaviors and poor prognosis in lung cancer. J Exp Clin Cancer Res.

[5] Cai S, Ye Z, Wang X, Pan Y, Weng Y, Lao S (2015). Overexpression of p21-activated kinase 4 is associated with poor prognosis in non-small cell lung cancer and promotes migration and invasion. J Exp Clin Cancer Res.

[6] Liu M, Zhou K, Huang Y, Cao Y (2015). The candidate oncogene (mcrs1) promotes the growth of human lung cancer cells via the mir-155-rb1 pathway. J Exp Clin Cancer Res.

[7] Hatakeyama S (2011). Trim proteins and cancer. Nat Rev Cancer.

[8] Niikura T, Hashimoto Y, Tajima H, Ishizaka M, Yamagishi Y, Kawasumi M (2003). A tripartite motif protein trim11 binds and destabilizes humanin, a neuroprotective peptide against alzheimer’s disease-relevant insults. Eur J Neurosci.

[9] Ishikawa H, Tachikawa H, Miura Y, Takahashi N (2006). Trim11 binds to and destabilizes a key component of the activator-mediated cofactor complex (arc105) through the ubiquitin-proteasome system. FEBS Lett.

[10] Tuoc TC, Stoykova A (2008). Trim11 modulates the function of neurogenic transcription factor pax6 through ubiquitin-proteosome system. Genes Dev.

[11] Hong SJ, Chae H, Lardaro T, Hong S, Kim KS (2008). Trim11 increases expression of dopamine beta-hydroxylase gene by interacting with phox2b. Biochem Biophys Res Commun.

[12] Di K, Linskey ME, Bota DA (2013). Trim11 is overexpressed in high-grade gliomas and promotes proliferation, invasion, migration and glial tumor growth. Oncogene.

[13] Qin Y, Cui H, Zhang H. Overexpression of trim25 in lung cancer regulates tumor cell progression. Technol Cancer Res Treat. 2015;9(1):23-45.10.1177/153303461559590326113559

[14] Khatamianfar V, Valiyeva F, Rennie PS, Lu WY, Yang BB, Bauman GS, Moussa M, Xuan JW. Trim59, a novel multiple cancer biomarker for immunohistochemical detection of tumorigenesis. BMJ Open. 2012;2(5):e001410.10.1136/bmjopen-2012-001410PMC348871923048060

[15] Huo X, Li S, Shi T, Suo A, Ruan Z, Yao Y (2015). Tripartite motif 16 inhibits epithelial-mesenchymal transition and metastasis by down-regulating sonic hedgehog pathway in non-small cell lung cancer cells. Biochem Biophys Res Commun.

[16] Li H, Zhang Y, Zhang Y, Bai X, Peng Y, He P (2014). Trim31 is downregulated in non-small cell lung cancer and serves as a potential tumor suppressor. Tumour Biol.

[17] Zhang YH, Wang Y, Yusufali AH, Ashby F, Zhang D, Yin ZF (2014). Cytotoxic genes from traditional chinese medicine inhibit tumor growth both in vitro and in vivo. J Integr Med.

[18] Chambers AF, Groom AC, MacDonald IC (2002). Dissemination and growth of cancer cells in metastatic sites. Nat Rev Cancer.

[19] Voulgari A, Pintzas A (2009). Epithelial-mesenchymal transition in cancer metastasis: Mechanisms, markers and strategies to overcome drug resistance in the clinic. Biochim Biophys Acta.

[20] Roberts PJ, Der CJ (2007). Targeting the raf-mek-erk mitogen-activated protein kinase cascade for the treatment of cancer. Oncogene.

[21] Vivanco I, Sawyers CL (2002). The phosphatidylinositol 3-kinase akt pathway in human cancer. Nat Rev Cancer.

[22] Yilmaz M, Christofori G (2009). Emt, the cytoskeleton, and cancer cell invasion. Cancer Metastasis Rev.

[23] Huber MA, Kraut N, Beug H (2005). Molecular requirements for epithelial-mesenchymal transition during tumor progression. Curr Opin Cell Biol.

[24] Yang J, Weinberg RA (2008). Epithelial-mesenchymal transition: At the crossroads of development and tumor metastasis. Dev Cell.

[25] Saharinen P, Eklund L, Pulkki K, Bono P, Alitalo K (2011). Vegf and angiopoietin signaling in tumor angiogenesis and metastasis. Trends Mol Med.

[26] Egeblad M, Werb Z (2002). New functions for the matrix metalloproteinases in cancer progression. Nat Rev Cancer.

[27] Johnson GL, Lapadat R (2002). Mitogen-activated protein kinase pathways mediated by erk, jnk, and p38 protein kinases. Science.

[28] Manning BD, Cantley LC (2007). Akt/pkb signaling: Navigating downstream. Cell.

[29] Fidler IJ (2003). The pathogenesis of cancer metastasis: The ‘seed and soil’ hypothesis revisited. Nat Rev Cancer.

[30] Tang JM, He QY, Guo RX, Chang XJ (2006). Phosphorylated akt overexpression and loss of pten expression in non-small cell lung cancer confers poor prognosis. Lung Cancer.

